The article "Acupuncture Improves Endometrial Angiogenesis by Activating PI3K/AKT Pathway in a Rat Model with PCOS" was published in 2022. Journal: Evid Based Complement Alternat Med.

# Acupuncture Improves Endometrial Angiogenesis by Activating PI3K/AKT Pathway in a Rat Model with PCOS

**DOI:** 10.1155/2022/1790041

**Published:** 2022-08-24

**Authors:** Liwei Xing, Yang Chen, Zhe He, Ming He, Yuhuan Sun, Jinlong Xu, Jian Wang, Haina Zhuang, Zeqin Ren, Ying Chen, Jun Yang, Shuluo Cheng, Rong Zhao

**Affiliations:** ^1^Yunnan University of Chinese Medicine, Kunming, China; ^2^Hainan Women and Children's Medical Center (Women and Children's Health Care Center of Hainan Province, Hainan Children's Hospital, Children's Hospital of Fudan University at Hainan, Hainan Obstetrics and Gynecology Hospital), Haikou, China; ^3^Yunnan Matemal and Child Health Care Hospital, Kunming, China; ^4^First Affiliated Hospital of Dali University, Dali, China; ^5^Nanjing Integrated Traditional Chinese and Western Medicine Hospital, Nanjing, China

## Abstract

**Background:**

Acupuncture, a treatment derived from traditional Chinese medicine, can effectively relieve the symptoms and improve pregnancy outcome in patients with polycystic ovary syndrome (PCOS); however, its mechanism remains unclear. This study aimed at investigating whether acupuncture could improve endometrial angiogenesis and thus endometrial receptivity via activating PI3K/AKT pathway in PCOS rats.

**Methods:**

We established a rat model with PCOS, which was induced by DHEA. Acupuncture was performed every other day for 15 days, and the PI3K inhibitor (LY294002) was intraperitoneal injected 30 mins before acupuncture treatment. Females rats were mated with male SPF SD rats in a ratio of 2 : 1 after treatment and sacrificed on the 5th day when the vaginal plug was identified. The number of implantation sites was observed, followed by ovarian and endometrial morphology detected with hematoxylin-eosin staining and a scanning electron microscope, estrous cycle detected with vaginal smear analysis, and sex hormones and angiogenesis-related PI3K/AKT gene/protein expression detected with enzyme-linked immunosorbent assay, western blotting, immune histochemistry, and quantitative real-time PCR.

**Results:**

Acupuncture notably improved implantation sites' number, endometrial receptivity factors including endometrial morphology, pinopodes, HOX-10, and LIF protein expression, as well as angiogenesis and PI3K/AKT pathway factors such as VEGF, VEGFR2, Ang-1, PI3K, AKT, and P-AKT gene/protein expression and the level of eNOS and NO in the endometrium of rats with PCOS; PCOS-like symptoms were alleviated as well. The efficacy of acupuncture on a rat model with PCOS was counteracted by the combination with the PI3K inhibitor.

**Conclusion:**

Acupuncture improves endometrial angiogenesis by activating the PI3K/AKT pathway, thus promoting endometrial receptivity and the number of implantation sites in rats with PCOS.

The article "Acupuncture Improves Endometrial Angiogenesis by Activating PI3K/AKT Pathway in a Rat Model with PCOS" was published in 2022. Journal: Evid Based Complement Alternat Med.

## 1. Introduction

Polycystic ovarian syndrome (PCOS) is a complex endocrine and metabolic disorder in gynecology and mainly characterized by hyperandrogenism and insulin resistance [1]. Up to 72% of patients with PCOS experience infertility, with the prevalence among women of reproductive age being 5–20% [2]. Infertility due to PCOS will exacerbate patients' psychological illnesses including anxiety, depression, and other mental health issues, which will eventually result in metabolic syndrome (obesity), type 2 diabetes, and cerebrovascular disorders [3]. Gonadotropin-releasing hormone agonist (GnRHa) or clomiphene (CC) is currently being used for PCOS, with ovulation rates of 50%, pregnancy rates of only 23.9%, and abortion rates of 25.8% [4]. Therefore, it is crucial to explore the effective methods alleviating a high ovulation rate and a low pregnancy rate in patients with PCOS.

Impaired endometrial receptivity (ER), which was induced by the dysfunction of cytokines, proteomics, and gene expression, is the major reason for low fertility as it prevents embryo implantation development in patients with PCOS [5]. The endometrial epithelium permits implantation during a brief period known as the implantation window (WOI) due to the endometrial receptivity [6]. Recently, studies have focused on angiogenesis together with increased vascular permeability, which were considered to be the key factors in endometrial decidualization, embryo implantation, and placentation. Vascular endothelial growth factor (VEGF) is a representative regulator of angiogenesis and vascular permeability [7]. Kodaman et al. reported that the increased expression of VEGF in the middle and late menstrual luteal periods was spatially synchronized with the WOI, which could be considered a molecular marker of ER [8–10]. Zhao et al. reported that VEGF mRNA and protein expression in PCOS endometrium decreased significantly at the WOI, which indicated impaired endometrium angiogenesis existed in patients with PCOS [11]. VEGF activates through the PI3K/AKT signaling pathway, which is the regulatory center for angiogenesis. Wang et al. reported that the expression of PI3K/AKT signaling pathway-related proteins was impaired during the WOI period of patients with PCOS [12]. Above all, we speculated the decreased endometrial receptivity induced by PI3K/AKT signaling pathway-mediated angiogenesis disorder was involved in the occurrence of infertility in PCOS.

Acupuncture is a traditional Chinese medicine without obvious side effects. A great deal of studies proved that acupuncture could effectively increase the pregnancy rate and relieve the symptoms of PCOS. Cheng's research suggested that acupuncture might increase the pregnancy rate of patients undergoing IVF-ET by the regulation of ncRNAs [13]. Xu's research suggested that acupuncture can break the vicious cycle initiated by excessive androgen secretion and regulate the androgen receptor as well as connexin 43 in PCOS to improve the reproductive function [14]. Studies reported that acupuncture can improve endometrial receptivity in superovulation mice via miR-494-3p/HOXA10 axis [15]. Our previous study revealed that angiogenesis disorder may be related to ER disorder during the WOI period in patients with PCOS due to the decreasing VEGF expression in the endometrium, while acupuncture can notably increase VEGF expression and improve endometrial thickness, morphology, blood perfusion, and endometrial receptivity, and ultimately pregnancy rates. Although the mechanism is yet unknown, few studies have examined the effectiveness of acupuncture in improving ER at the WOI stage; in addition, the study focused on the endometrial PI3K/AKT pathway during the WOI period in patients with PCOS. The majority of previous studies mostly focused on follicular growth and the proliferation of ovarian granulosa cells in PI3K/AKT and angiogenesis pathways. We hypothesized that acupuncture can improve endometrial angiogenesis by activating the PI3K/AKT pathway, thus promoting endometrial receptivity in rats with PCOS.

The article "Acupuncture Improves Endometrial Angiogenesis by Activating PI3K/AKT Pathway in a Rat Model with PCOS" was published in 2022. Journal: Evid Based Complement Alternat Med.

In this study, a PCOS-like rat model was established by dehydroepiandrosterone (DHEA) injection. Acupuncture-mediated modulation of the PI3K/AKT signaling pathway and its involvement in PCOS-like symptoms, endometrial receptivity, implantation sites' number, and angiogenesis were further investigated. Our findings shed light on the novel protective mechanisms of acupuncture in treating PCOS.

## 2. Materials and Methods

### 2.1. Animal Modeling and Grouping

Forty-five three-week-old female Sprague-Dawley (SD) rats were purchased from Hunan SJA Laboratory Animal Co, Ltd. (Hunan, China). Thirty-five female SPF SD rats were randomly selected to establish the PCOS model. Of these rats, 30 established PCOS models verified from the body weight, ovarian pathology, estrous cycle, and sex hormone levels were randomly divided into the model group (model), the acupuncture group (Acu), and the PI3K inhibitor + acupuncture group (PI + Acu) (*n* = 10 per group). In addition, 10 female SPF SD rats were selected as the normal control group (control). The PCOS model was induced by daily subcutaneous injection with DHEA (Biotopped, China) at a dose of 6 mg/100 g body weight and sesame oil (Liaoning Shinsun Pharmaceutical Co., Ltd, China) at a dose of 0.2 ml/d for 20 consecutive days [16]. After verifying the establishment of the PCOS model, appropriate treatment was initiated in each group. Acupuncture treatment was performed every other day for 15 days. According to our previous study [17–19], the acupuncture points SP4, PC6, EX-CA1, and CV4 will be selected. Huatuo milli-needles (0.19 mm × 10.00 mm, Suzhou Medical Equipment Co., Ltd.) were inserted perpendicularly or obliquely into the abovementioned acupuncture points, the depth of which was 3 mm. The acupuncture duration was 20 min every time. The rats in the PI + Acu group received intraperitoneal injection with 0.3 mg/kg LY294002 (Abcam, UK) at 30 min before each acupuncture treatment [20]. The rats in the control and model groups were received intragastric administration with saline. Saline treatment was performed every other day for 15 days.

The article "Acupuncture Improves Endometrial Angiogenesis by Activating PI3K/AKT Pathway in a Rat Model with PCOS" was published in 2022. Journal: Evid Based Complement Alternat Med.

### 2.2. Sample Collection

After 15 days' treatment, the female rats were mated with male SPF SD rats in a ratio of 2 : 1. Rats were sacrificed during the implantation window time on the 5th day when the vaginal plug was identified. Rats were anesthetized with 3% pentobarbital sodium (0.1 ml/100 g of body weight), and then, blood samples were obtained from the abdominal aorta after overnight fasting. Blood samples were then centrifuged at 3000g for 15 min at 4°C for ELISA. The whole uteri from 5 random rats of each group were collected for implantation sites' number and SEM examination. The collection of endometria from the other 5 random rats of each group was divided into five parts: one for HE and four for gene and protein expression analysis using immunohistochemistry, ELISA, qRT-PCR, and western blot, respectively. The ovarian tissue will also be collected for HE detection.

### 2.3. Weighing

Body weight was measured every 2 days from the first day of DHEA subcutaneous injection. The last weighing was carried out at the time of sample collection. The ovary wet weight was measured, and the ovarian index was calculated after the rats were sacrificed. Body weight gain = (weight of rats before sacrifice-initial weight)/initial weight × 100%. Ovarian index = ovarian wet weight/body weight.

### 2.4. Vaginal Smear Analysis

Vaginal smear analysis was performed daily at 9 am from 10 days after DHEA treatment. Vaginal cells were collected via saline lavage and dropped onto a glass slide. After air-drying, they were stained with 0.1% methylene blue (Solarbio, China). Estrous stages were determined based on the predominant cell type as described previously [21].

### 2.5. Implantation Sites' Number Examination

The whole uteri dissection was performed rapidly on ice and collected for implantation sites' number. After removing fat and the connective tissue, the uteri were separated and the conceptuses were removed. The number of implantation sites was recorded.

The article "Acupuncture Improves Endometrial Angiogenesis by Activating PI3K/AKT Pathway in a Rat Model with PCOS" was published in 2022. Journal: Evid Based Complement Alternat Med.

### 2.6. Enzyme-Linked Immunosorbent Assay (ELISA)

Rat serum sex hormones (T, E2, LH, FSH) and eNOS and NO in the endometrium of the rat were measured with an ELISA kit (MEIMIAN, Yancheng, China) according to the manufacturer's instructions. Briefly, the assay was applied to rat serum in a 96-well low-adherent white-luminescent plate. First, diluent sample of 100 *μ*l was infused into the corresponding pore of an enzyme scale plate, gently mixed for 30 s, and incubated for 90 min at 37°C. Second, we discarded all of the liquid in the enzyme scale plate, washed the enzyme scale plate with eluent, and removed the water with drying paper. The washing and drying were repeated three times. Subsequently, 100 *μ*l of enzyme-labeling reagent was added to each pore, except for the blank pore, and incubated for 30 min at 37°C away from light; the washing and drying were repeated five times. Thereafter, the enzyme-labeling reagent was replaced with 50 *μ*l each of chromogenic agents A and B, and the plate was gently mixed for 10s and incubated for 15 min at 37°C away from light. Stop buffer was added, and the solution was gently mixed for 30 s. Each pore's OD value was then measured at 450 nm with a spectrophotometer within 15 min of the addition of stop solution.

### 2.7. Hematoxylin-Eosin (H&E) Staining

After fixation in 4% paraformaldehyde, the ovaries and uterus were embedded in paraffin, and 4-*μ*m serial sections were produced. The sections were mounted on slides and immersed in xylene (10 min, twice) and rehydrated in a decreasing ethanol series diluted in distilled water (100%, 100%, 95%, 90%, 80%, and 70%, 1 min each). The sections were then rinsed in deionized water, stained in hematoxylin for 80 s, rinsed in deionized water, and finally stained in eosin for 3 s. After the color reaction, the sections were dehydrated through an ethanol series in xylene. The sections were taken using an IX73 microscope (Olympus Corporation, Japan). ImageJ (Image in Java, USA) software was used to observe the morphology of ovary, determine the thickness of the endometrium (the vertical distance from the endometrial junction to the myometrium to the uterine cavity), and calculate the number of blood vessels in three different fields of view, with their averages recorded.

### 2.8. Scanning Electron Microscope (SEM)

Ultrastructural changes of pinopodes in the endometrium were observed using the BA600Mot scanning electron microscope (SEM) (MOTIC, Canada). Briefly, the endometrium tissues were prefixed with 2.5% glutaraldehyde. Following this, they were dehydrated with acetone and soaked in isoamyl acetate for 2 h. Then, vacuum drying and metal coating were used for the tissue treatment. The treated tissues were observed by SEM.

The article "Acupuncture Improves Endometrial Angiogenesis by Activating PI3K/AKT Pathway in a Rat Model with PCOS" was published in 2022. Journal: Evid Based Complement Alternat Med.

### 2.9. Immunohistochemistry (IHC)

Samples were fixed with fresh 4% paraformaldehyde and underwent conventional histological procedures for embedding in paraffin. These samples were cut into 4.5-*μ*m-thick sections, processed for IHC staining with anti-VEGF polyclonal antibody (GB11034B, Servicebio, China) and rabbit anti-Ang-1 polyclonal antibody (ab95230, Abcam, UK), and then incubated with secondary antibodies. The images were digitized by fluorescence microscopy using an IX73 microscope (Olympus Corporation, Japan). The positive cells' density of each slice was measured by image analysis software Image-Pro Plus 6.0.

### 2.10. Western Blotting

Total protein was extracted from endometrium tissues using RIPA buffer (Servicebio, China) supplemented with 1% PMSF (Servicebio, China). Protein quantification was performed using an Enhanced BCA Protein Assay Kit (Servicebio, China). Sodium dodecyl sulfate polyacrylamide gel electrophoresis was carried out for protein separation. Then, the protein samples were transferred onto the PVDF membrane (Servicebio, China) and blocked in 5% BSA (Servicebio, China). Subsequently, the membranes were incubated with the primary antibodies against HOXA10 (ab191470, Abcam, UK), LIF (ab138002), VEGF (GB11034B, Servicebio, China), VEGFR2 (GB11190, Servicebio, China), P-PI3K (GB11190, Servicebio, China), AKT (GB111114, Servicebio, China), P-AKT (AF3242, Affinity, USA), and ACTIN (GB15001, Servicebio, China) at 4°C overnight. After washing with TBS-T three times, the membranes were then incubated with the secondary antibody at RT for 1h and detected using an ECL plus kit (G2019, Servicebio, China). PhotoShop software (alphaEaseFC, Alpha Innotech, USA) was used to remove the color, and Alpha software (Adobe PhotoShop, Adobe, USA) was used to analyze the optical density of the target band.

### 2.11. Quantitative Reverse Transcription-Polymerase Chain Reaction (qRT-PCR)

Total RNA was extracted from the harvested uteri using the TRIzol reagent (Gibco), and 1 *μ*g of total RNA was subjected to the reverse transcription of mRNA using oligo dT as a primer and a reverse transcription kit (Servicebio, Wuhan, China) to generate total cDNA. A quantitative PCR was then carried out using the primers shown in Table 1 and a fluorescence ration PCR instrument (Bio-Rad, California, USA). R-Actin was used for normalization. The quantitative expression level was analyzed using the 2^−ΔΔCt^ method.

The article "Acupuncture Improves Endometrial Angiogenesis by Activating PI3K/AKT Pathway in a Rat Model with PCOS" was published in 2022. Journal: Evid Based Complement Alternat Med.

### 2.12. Statistical Analysis

Data analysis was performed with SPSS 26.0 software. The data were expressed as means ± standard deviation (SD). The means and SD were calculated from three independent experiments. Student's *t*-test was used to compare the differences between two groups. One-way analysis of variance (ANOVA) was used for comparisons between multiple groups. *P* < 0.05 was considered to be statistically significant.

## 3. Results

### 3.1. Inhibition of PI3K/AKT Pathway Reversed the Beneficial Effect of Acupuncture on Rats with PCOS

As shown in Figures 1(a) and 1(b), the body weight gain and the ovarian index in the model group were much higher than those in the control group (*P* < 0.05). The body weight gain and the ovarian index of the acupuncture group were lower than those in the model group (*P* < 0.05). However, the PI3K inhibitor reversed the effect of acupuncture on weight gain and the ovarian index (*P* < 0.05)

In addition, SD rats have an estrous cycle of about 4-5 days. The vaginal smear results of the rats are shown in Figure 1(c). The vaginal smear in the proestrus stage is mainly composed of nuclear epithelial cells (NE, the red arrows). The estrous stage is mainly composed of epithelial keratinocytes (EK, the green arrows). Leukocytes (L, the black arrows) and nuclear epithelial cells are the main components at the metestrus stage with keratinocytes occasionally. The diestrus stage is almost entirely leukocytes. Figures 1 1-1, 1-2, 1-3, and 1-4 are the vaginal smears of rats in the control group on days 1 to 4. 1-1: The proestrus stage is mainly composed of nuclear epithelial cells; 1-2: the estrous stage is mainly composed of epithelial keratinocytes; 1-3: leukocytes and nuclear epithelial cells are the main components at the metestrus stage with keratinocytes occasionally; 1-4: the diestrus stage is almost entirely leukocytes. In the Acu group, there was a complete estrous cycle as the control group (3-1, 3-2, 3-3, and 3-4 same as 1-1, 1-2, 1-3, and 1-4). But in the model and PI + Acu groups, 2-1, 4-1 are at the vaginal smear during the metestrus stage (same as 1-3); 2-2, 4-2 are at the vaginal smear during the metestrus stage (same as 1-3); 2-3, 4-3 are at the vaginal smear during the proestrus stage (same as 1-1); and 2-4, 4-4 are at the vaginal smear during the proestrus stage (same as 1-1). In our research, we discovered that the control group experienced a full estrous cycle. The model group experienced the estrous cycle abnormality almost at the proestrus and metestrus stages. Anovulation is a sign that there is no estrus. The acupuncture group's estrous cycle steadily improved. The inhibition of PI3K/AKT caused by PI3K inhibitors undid the effects of acupuncture on the typical estrous cycle.

The article "Acupuncture Improves Endometrial Angiogenesis by Activating PI3K/AKT Pathway in a Rat Model with PCOS" was published in 2022. Journal: Evid Based Complement Alternat Med.

Moreover, as shown in Figure 1(d), the serum levels of E2, T, LH, and LH/FSH ratio in model rats detected by ELISA were remarkably elevated compared to control rats, while the serum P and FSH levels were reduced by almost half, whereas these changes were attenuated by acupuncture intervention. Effects of acupuncture were reversed by the PI3K inhibitor.

Besides, the results of HE staining of ovary tissue were presented in Figure 1(e). In the control group, the ovarian tissue from the control group had a normal appearance. Different stages of ovarian follicles, multilayer follicle granulosa cells (8-9 layers), oocytes, and corona in follicles were observed. While the number of atretic follicles and cystic dilating follicles increased significantly with fewer layers of granular cells, there is a lack of oocytes and corona radiating within the follicles in the model group. The corpus luteum was significantly reduced. The ovarian tissue from the acupuncture group showed increased granular cell layers and some ovulation phenomena. After a combination intervention of acupuncture and the PI3K inhibitor, the number of atretic follicles and cystic dilating follicles increased significantly with fewer layers of granular cells, and there is a lack of oocytes and corona radiating within the follicles. The above results suggested that compared with the control and acupuncture groups, the number of atretic follicles and cystic dilating follicles increased significantly with fewer layers of granular cells, and there is a lack of oocytes and corona radiating within the follicles. The corpus luteum was significantly reduced. DHEA-induced increased atretic follicles and cystic dilating follicles were relieved by acupuncture intervention; however, the PI3K inhibitor counteracted the therapeutic effect of acupuncture.

### 3.2. Inhibition of PI3K/AKT Pathway Reversed the Acupuncture-Mediated Changes in Implantation Sites Number and Endometrial Receptivity on Rats with PCOS

We further investigated the effectiveness of acupuncture in implantation sites' number and endometrial receptivity, as well as the involvement of the PI3K/AKT pathway in acupuncture-mediated changes, since a decreased implantation site number and endometrial receptivity are two of the key pathological features of PCOS. As can be seen from Figure 2(a), there were fewer implantation sites in the model group as compared to the control group (*P* < 0.05). The number of implantation sites was shown to be increased in the acupuncture group; however, *P* < 0.05. The reduction in the number of implantation sites caused by acupuncture was reversed by the inhibition of PI3K/AKT by the PI3K inhibitor.

The article "Acupuncture Improves Endometrial Angiogenesis by Activating PI3K/AKT Pathway in a Rat Model with PCOS" was published in 2022. Journal: Evid Based Complement Alternat Med.

Furthermore, the endometrial structure in the control group was intact, the epithelial cells were neatly aligned, and the blood vessels and glands were clearly apparent from the HE scans, as shown in Figure 2(b). The endometrial glands and blood arteries were in scarce in the model group, and there was obvious significant endometrial thinning. The endometrial thicknesses in the acupuncture group (*P* < 0.05) considerably increased as compared to the model group. The acupuncture group also experienced an increase in endometrial blood vessels. However, acupuncture's healing effects were negated by PI3K inhibitors. In addition, the endometrial pinopodes detected by SEM shown in Figure 2(c) showed that there were a major number of pinopodes on the surface of endometrium in the control and acupuncture groups, while few pinopodes can be found in the model group. An acupuncture-mediated increase in pinopodes was significantly repressed by combination with the PI3K inhibitor.

HOXA10 and LIF, indicators of endometrial receptivity, were also shown to be expressed by western blotting, as shown in Figure 2(d). According to the western blotting results, both the control group and the acupuncture group had significantly higher levels of HoxA10 and LIF expression as compared to the model group. HoxA10 and LIF expression changes brought on by acupuncture, however, were reversed when PI3K/AKT was inhibited by the PI3K inhibitor.

### 3.3. Inhibition of PI3K/AKT Pathway Reversed the Acupuncture-Mediated Changes in Endometrial Angiogenesis on Rats with PCOS

Since the PI3K/AKT pathway is an important representative of angiogenesis, next, we investigated the improvement in endometrial angiogenesis underlying the beneficial effects of acupuncture on PCOS and the involvement of the PI3K/AKT pathway in acupuncture-mediated changes. As shown in Figure 3(a) which was detected by IHC, the localization of VEGF was observed in an IHC analysis. The cytoplasm of vascular endothelial cells, mesenchymal cells, and endometrial glandular epithelial cells all expressed VEGF protein and displayed brownish yellow granules. The findings demonstrated that the model group's VEGF-positive cell density was significantly lower than that of the control group (*P* < 0.05). Following acupuncture, the endometrial tissue displayed a brown-yellow particle accumulation with positive staining. The acupuncture group had a higher density of positive cells than the model group did. In contrast, the combination of a PI3K inhibitor and acupuncture greatly reduced the increase in VEGF caused by acupuncture.

The article "Acupuncture Improves Endometrial Angiogenesis by Activating PI3K/AKT Pathway in a Rat Model with PCOS" was published in 2022. Journal: Evid Based Complement Alternat Med.

According to Figure 3(b), immunohistochemistry examination revealed that the majority of the perivascular matrix contained Ang-1, which presented brownish yellow granules, suggesting that Ang-1 promoted angiogenesis by acting on the blood vessels. The findings demonstrated that the model group's positive Ang-1 cell density was significantly lower than that of the control group (*P* < 0.05). When compared to the model group, the acupuncture group experienced a substantial increase in brown-yellow particle deposition with positive staining (*P* < 0.05). In contrast, the combination of a PI3K inhibitor and acupuncture greatly suppressed the increase in Ang-1 caused by acupuncture.

### 3.4. Effect of Acupuncture on PI3K/AKT Pathway Expression in Rats with PCOS

Since PI3K/AKT pathway promotion participated in the protection of acupuncture against PCOS in PCOS-like symptoms, implantation sites' number, endometrial receptivity, and endometrial angiogenesis, the regulation of acupuncture in PI3K/AKT pathway expression was further investigated in PCOS rats. As presented in Figure 4(a), the western blotting results showed that as compared to the model group, the expression of VEGF, VEGFR2, P-PI3K, AKT, and P-AKT in the endometrium tissue were upregulated in the acupuncture group with a significant increase, whereas an acupuncture-mediated increase in VEGF, VEGFR2, AKT, P-PI3K, and P-AKT was repressed by combination with the PI3K inhibitor. Compared with the acupuncture group, the levels of VEGF, VEGFR2, P-PI3K, AKT, and P-AKT in the PI3K inhibitor + acupuncture group were significantly decreased.

As shown by the results of the qRT-PCR of *Vegf*, *Vegfr*, *Pi3k*, and *Akt* expression in the endometrium at the mRNA level in Figure 4(b), *Vegf*, *Vegfr*, *Pi3k,* and *Akt* mRNA levels were reduced in the model group as compared to the control group (*P* < 0.05). In contrast, the upregulated expression of *Vegf*, *Vegfr*, *Pi3k*, and *Akt* mRNA was detected in the acupuncture group (*P* < 0.05). The suppression of PI3K/AKT by the PI3K inhibitor reversed acupuncture-mediated changes in *Vegf*, *Vegfr*, *Pi3k*, and *Akt* mRNA levels.

Since eNOS and NO are important molecules of the PI3K/AKT signaling pathway, we detected the expression of eNOS and NO in uterine tissues by ELISA. As shown in Figure 4(c), the endometrial tissue eNOS and NO expression in model rats was remarkably reduced compared to control rats (*P* < 0.05). However, these changes were attenuated by acupuncture intervention. Effects of acupuncture were reversed by the PI3K inhibitor.

## 4. Discussion

PCOS, a complex disease of reproductive endocrine system, is the main cause of infertility. Reduced endometrial receptivity caused by angiogenesis abnormalities may lead to a high abortion rate and a low implantation rate in patients with PCOS. A majority of studies suggested that acupuncture can improve ER and angiogenesis effectively in women with PCOS [22, 23]. However, the potential mechanisms of acupuncture underlying the efficacy of PCOS have not been fully illuminated.

The article "Acupuncture Improves Endometrial Angiogenesis by Activating PI3K/AKT Pathway in a Rat Model with PCOS" was published in 2022. Journal: Evid Based Complement Alternat Med.

Previous studies have demonstrated that the DHEA-induced rat model in PCOS displays the clinical characteristics of PCOS in humans, including hyperandrogenism, obesity, and pathological morphology of polycystic ovary [24]. Yu et al. indicated that decreased endometrial receptivity and abnormal ovarian morphology existed in mice exposed by DHEA [25]. Therefore, a rat model of PCOS induced by DHEA was established in the study, which showed typical PCOS-like symptoms like considerable increases in body weight and ovarian index, disruption of the estrous cycle, abnormal sex hormone levels, and abnormal ovarian morphology, in line with the previous study [26]. According to previous studies, acupuncture can relieve PCOS-like symptoms by balancing the levels of sex hormones and autophagy in ovarian tissues via regulating PI3K/AKT pathway [27]. In our study, acupuncture-induced alleviation in PCOS-like symptoms can be reversed by the PI3K inhibitor, indicating the PI3K/AKT pathway may be involved in the mechanism of acupuncture in PCOS, which is consistent with previous studies. Acupuncture can also control weight gain in rats with PCOS effectively due to the regulation of lipid metabolism and insulin resistance. Our earlier study suggested that acupuncture decreased leptin resistance by boosting the number of leptin receptors in the hypothalamus, altering the architecture of fat, and controlling blood lipid levels, which led to weight loss [28].

SP4, PC6, EX-CA1, and CV4 were selected due to their effectiveness in acupuncture-mediated treatment and for further investigation underlying the mechanism of acupuncture on patients with PCOS. Acupuncture points, SP4, PC6, EX-CA1, and CV4, were curative in ER-improving in patients with PCOS, as well as gonadal hormone concentrations and clinical pregnancy rate according to our previous study [17–19]. In the theory of traditional Chinese medicine, SP4 is luo-connecting point of spleen meridian, which can tonify qi and replenish blood, as well as promote local angiogenesis in the endometrium [29]. PC6 is luo-connecting point of the pericardium meridian, which can promote blood circulation to remove blood stasis [30]. EX-CA1 is a local point selection, which can increase endometrial vascular permeability and CV4 is point of conception vessel, which has effect on pregnancy and PCOS [31]. Some studies suggested that forementioned acupoints can regulate the hypothalamic-pituitary-ovarian axis bidirectionally and thus restore the secretion of FSH, LH, and E2 in patients with PCOS [32]. Also the clinical pregnancy rate was elevated by acupuncture on the above acupoints of patients with PCOS as well, whose molecular mechanism may be related to the expression of HOXA10, LIF, and some other endometrial receptivity factors [33].

The article "Acupuncture Improves Endometrial Angiogenesis by Activating PI3K/AKT Pathway in a Rat Model with PCOS" was published in 2022. Journal: Evid Based Complement Alternat Med.

Defected endometrial receptivity will lead to a reduced pregnancy rate due to endometrial epithelial cell attachment failure or poor embryo reception, which indicates that endometrial receptivity is crucial for embryo implantation [34]. The endometrial epithelium permits implantation during a brief period known as the implantation window (WOI) due to the endometrial receptivity [6]. And the characteristic pathology of PCOS, such as hyperandrogenemia, inflammation, insulin resistance, and obesity, can all result in the forementioned disorder [35]. Dechaud et al. reported that when the endometrial thickness ≤7 mm, the endometrial receptivity and pregnancy rate decreased, which implied endometrial thickness as an indicator to predict endometrial receptivity [36]. Liu considered blood vessel numbers as representative marker of blood supplement in endometrium [37]. Pinopodes, a smooth projection on the endometrial epithelium's membrane tip, are spatiotemporally synchronized with endometrial receptivity and as a morphological indicator of excellent endometrial receptivity [38]. HOXA10 is a crucial regulator of embryo implantation, controlling the expression of downstream genes to alter endometrial decidualization and embryo adhesion [39]. LIF is a pleiotropic cytokine that affects blastocyst implantation by encouraging the development of endometrial receptors and is directly targeted at endometrial epithelial cells [40]. In our study, the rat model with PCOS showed considerably fewer implantation sites, thinner endometrium thickness, fewer blood vessels, and pinopodes in the endometrium with lower levels of HOXA10 and LIF protein, all of which indicated defected endometrial receptivity in PCOS, while acupuncture can enhance the endometrial receptivity-related indicators mentioned above. As previous study mentioned before, acupuncture can prominently improve endometrial receptivity by different ways. You et al. reported that electroacupuncture could improve the endometrial receptivity and promote the blastocyst implantation in COH rats by reducing cell adhesion molecules and enhancing the LIF/STAT3 signaling pathway [41]. Also, significantly increased embryo implantation, endometrial thickness, numbers of glands, and blood vessels were observed in the acupuncture group, as well as significantly higher expression levels of pinopode-related markers, including integrin v3, homeobox A10 (HOXA10), heparin-binding EGF-like growth factor (HBEGF), estrogen receptor alpha (ER), and progesterone receptor (PR), which indicates that EA had a positive effect on the endometrial receptivity of thin endometrium model rats by improving pinopode formation through multiple molecular targets according to Xi's study [42]. Endometrial receptivity factors including endometrial morphology, pinopodes, HOX-10, and LIF protein expression were elevated after acupuncture in rats with PCOS detected by our study, which indicates that there is a notably curative effect of acupuncture on promoting endometrial receptivity in rats with PCOS.

The article "Acupuncture Improves Endometrial Angiogenesis by Activating PI3K/AKT Pathway in a Rat Model with PCOS" was published in 2022. Journal: Evid Based Complement Alternat Med.

Angiogenesis is the fundamental connection strongly tied embryo implantation and endometrial receptivity together [43]. Angiogenesis of the endothelial function layer and capillary epithelium in the early stages of endometrial proliferation and secretion, along with increased vascular endothelial growth factor and angiogenesis-related factor expression, leads to the thickening of the intima layer and subsequent growth of curly spiral artery, and makes the lining after ovulation and the implantation window receptively, which are prepared for embryo implantation [44]. Endometrial Ang-2 blocks Tie-2 signaling pathways with increased angiogenesis-related factor expression and exposes vascular epithelial cells, stromal cells, cell solution, and initial angiogenic factor recognition sites to endothelial surface; thus, angiogenesis is promoted with increased endometrial implant site blood perfusion during the budding stage, and endometrium decidualizes quickly when prepared for pregnancy [45]. VEGF and Ang have an impact on angiogenesis, which are key indicators for ER evaluation [46]. The process of the blastocyst on apposition, adhesion attachment, invasion penetration, and decidualization is ensured by VEGF, one of the earliest contacting-endometrium genes, which was activated at the point of implantation [44]. Ang-1 is strongly expressed in the endometrium during the embryo implantation period, which modulates the angiogenesis and is crucial for the successful implantation of blastocysts [47]. The immunohistochemical results in our study revealed that decreased levels of VEGF and ANG-1 existed in the endometrium of rats with PCOS rats, which was significantly elevated after acupuncture treatment, indicating that acupuncture can treat endometrial angiogenesis disorders brought on by PCOS in WOI.

The PI3K/AKT pathway is the center of regulation for angiogenesis, which controls endothelial cell survival, proliferation, and vascular permeability [48]. VEGF binding to VEGFR-2 will activate the release of NO by endothelial cells and ultimately trigger eNOS. eNOS and NO are indicators of vascular permeability and angiogenesis, which indicates that the PI3K/AKT pathway is tightly linked to angiogenesis and permeability. P-PI3K and P-AKT represent the activation of the PI3K/AKT pathway. When combining with the PI3K inhibitor, acupuncture-mediated improvements in PCOS-like symptoms, endometrial receptivity, the number of implantation sites, and endometrial angiogenesis were altered, indicating that the PI3K/AKT signaling pathway may be involved in the mechanism of acupuncture on rats with PCOS. As a result, we detected acupuncture's impacts on PI3K/AKT pathway-related proteins and mRNA expression. The results demonstrated that acupuncture dramatically enhanced the expression of VEGF, VEGFR2, P-PI3K, AKT, P-Akt protein and VEGF, VEGFR, PI3K, and AKT mRNA in the endometrium of PCOS rats, along with the rising of vascular permeability factors eNOS and NO. Acupuncture-induced alterations in the expression of the PI3K/AKT signaling pathway were, however, restored by PI3K inhibitors. Notably, P-PI3K and P-AKT protein expression by WB and PI3K, and AKT mRNA expression by qRT-PCR were considerably lower in the PI + Acu group compared to the Acu group. It has been proposed that the phosphorylation, or activation, of the PI3K/AKT pathway may be connected to the mechanism of acupuncture. According to previous studies, P-PI3K and P-Akt total protein expression were significantly higher in the endometrium of women who were successfully pregnant during the WOI stage compared to the other stages, indicating that the PI3K/AKT signaling pathway is activated and may play a role in the development of endometrial receptivity and pregnancy [49].

The article "Acupuncture Improves Endometrial Angiogenesis by Activating PI3K/AKT Pathway in a Rat Model with PCOS" was published in 2022. Journal: Evid Based Complement Alternat Med.

As a result, our study demonstrated that acupuncture notably improved the implantation sites' number, endometrial receptivity factors including endometrial morphology, pinopodes, HOX-10, and LIF protein expression, as well as angiogenesis and PI3K/AKT pathway factors such as VEGF, VEGFR2, Ang-1, PI3K, AKT, P-AKT gene/protein expression, and the level of eNOS and NO in the endometrium of rats with PCOS; PCOS-like symptoms were alleviated as well. The efficacy of acupuncture on the rat model with PCOS was counteracted by the combination with the PI3K inhibitor.

The above results indicate that acupuncture improves endometrial angiogenesis by activating the PI3K/AKT pathway, thus promoting endometrial receptivity and the number of implantation sites in PCOS rats, as illustrated in Figure 5.

## 5. Conclusion

Taken together, our findings indicate that acupuncture improves endometrial angiogenesis by activating the PI3K/AKT pathway, thus promoting endometrial receptivity and the number of implantation sites in PCOS rats. Our study provides novel insight into the mechanisms underlying the treatment of acupuncture in PCOS, which offers more theoretic foundation for its clinical application.

## Figures and Tables

**Figure 1:** Inhibition of the PI3K/AKT pathway reversed the beneficial effect of acupuncture on rats with PCOS. (a) Body weight gain. (b) Ovarian index. (c) Cycle detection by vaginal smear analysis (×200). Red arrow: nuclear epithelial cell (NE). Green arrow: epithelial keratinocyte (EK). Black arrows: leukocyte L. (d) Sex hormones by ELISA. (e) H&E staining of the rat ovary tissue (×100). AF: atretic follicle, CF: cystic follicle, CR: corona radiate, GCL: granular cell layer, L luteal, O oocyte, TCL: theca cell layer. Control: the control group; model: the model group; Acu: the acupuncture treatment group; and PI + Acu: the PI3K inhibitor combined with the acupuncture treatment group. ^*∗*^*P* < 0.05 as compared to the control group; ^#^*P* < 0.05 as compared to the model group; ^△^*P* < 0.05 as compared to the acupuncture group.

**Figure 2:** Inhibition of the PI3K/AKT pathway reversed the acupuncture-mediated changes in blastocysts number and endometrial receptivity on rats with PCOS. (a) The number of blastocysts. (b) H&E staining of rat uterine tissue (×40, ×100). Arrows: endometrial thickness. Endometrial thicknesses and blood vessels in each group. (c) Ultrastructural changes of endometrial pinopodes by SEM (x5000). (d) WB results and the histograms of western blot analysis for HOXA10 and LIF. Control: the control group; Model: the model group; Acu: the acupuncture treatment group; and PI + Acu: the PI3K inhibitor combined with the acupuncture treatment group. ^*∗*^*P* < 0.05 as compared to the control group; ^#^*P* < 0.05 as compared to the model group; ^△^*P* < 0.05 as compared to the acupuncture group.

**Figure 3:** Inhibition of the PI3K/AKT pathway reversed the acupuncture-mediated changes in endometrial angiogenesis on rats with PCOS. (a) VEGF protein expression by IHC (×400). (b) Ang-1 protein expression by IHC (×400). Arrows: the site where brown-yellow particles were deposited. Control: the control group; model: the model group; Acu: the acupuncture treatment group; and PI + Acu: the PI3K inhibitor combined with the acupuncture treatment group. ^*∗*^*P* < 0.05 as compared to control group; ^#^*P* < 0.05 as compared to the model group; ^△^*P* < 0.05 as compared to the acupuncture group.

The article "Acupuncture Improves Endometrial Angiogenesis by Activating PI3K/AKT Pathway in a Rat Model with PCOS" was published in 2022. Journal: Evid Based Complement Alternat Med.

**Figure 4:** Effect of acupuncture on PI3K/AKT pathway expression in rats with PCOS. (a) WB results and the histograms of western blot analysis for VEGF, VEGFR2, P-PI3K, AKT, and P-AKT. (b) qRT-PCR result of VEGF, VEGFR2, PI3K, and AKT mRNA expression. Control: the control group; model: the model group; Acu: the acupuncture treatment group; and PI + Acu: the PI3K inhibitor combined with the acupuncture treatment group. ^*∗*^*P* < 0.05 as compared to the control group; ^#^*P* < 0.05 as compared to the model group; ^△^*P* < 0.05 as compared to the acupuncture group.

**Figure 5:** Mechanism of acupuncture improving endometrial angiogenesis by activating the PI3K/AKT pathway in PCOS rats.

**Table 1:** Primers for qRT-PCR.

Gene name	Primer sequence
R-*Gapdh*-S	CTGGAGAAACCTGCCAAGTATG
R-*Gapdh*-A	GGTGGAAGAATGGGAGTTGCT
R-*Vegf* (2)-S	TGTGAGCCTTGTTCAGAGCG
R-*Vegf* (2)-A	GGTCTAGTTCCCGAAACCCTGA
R-*Vegfr*2 (4)-S	CAAGTCCGAATCCCTGTGAAGT
R-*Vegfr*2 (4)-A	GGTGAGGATGACCGTGTAGTTTC
R*-Pi3k* (5)-S	CCTGGTGATTGAGAAGTGTAAAGTG
R*-Pi3k* (5)-A	CGTAAGGCAGAAGGCACAGGT
R-*Akt* (4)-S	CTGGAGGACAACGACTATGGC
R-*Akt* (4)-A	AGCCTCTGTGTAGGGTCCTTCTT

## Data Availability

The data used to support the findings of this study can be obtained from the corresponding author upon request.
